# Comparative Gross Anatomy of the Forelimb Arteries of the Japanese Monkey (*Macaca fuscata*) and a Comparative Pattern of Forelimb Arterial Distribution in Primates

**DOI:** 10.1155/2020/8635917

**Published:** 2020-07-15

**Authors:** Tales Alexandre Aversi-Ferreira, Emmanuel Freitas-Ferreira, Roqueline A. G. M. F. Aversi-Ferreira, Karolyne Cordeiro-de-Oliveira, Gezianne Lopes-de-Freitas, Kaynara Trevisan, Giovanna Felipe Cavalcante, Ediana Vasconcelos-da-Silva, Sylla Figueredo-Silva, Renata Cristina Pereira, Dyecika Souza Couto, Rosângela Correa Rodrigues, Tainá de Abreu

**Affiliations:** ^1^Laboratory of Biomathematics and Physical Anthropology, Department of Structural Biology, Institute of Biomedical Sciences, Federal University of Alfenas, Alfenas, Minas Gerais, Brazil; ^2^School of Nutrition, Federal University of Alfenas, Alfenas, Minas Gerais, Brazil; ^3^Laboratório de Psicofisiologia Sensorial, Departamento de Psicologia Experimental, Universidade de São Paulo-USP, São Paulo, São Paulo, Brazil; ^4^Palmas' College (FAPAL), Nursing Course Coordination, Palmas, Tocantins State, Brazil; ^5^Museum of Morphology, Federal University of Tocantins, Palmas, Brazil; ^6^Department of Biological Sciences, State University of Feira de Santana, Feira de Santana, Bahia, Brazil

## Abstract

*Macaca fuscata* displays characteristic behaviours, such as stone handling, locomotor behaviour, gait position, and intermittent bipedalism. Differences in characteristic behaviours among primate species/genera could be explained by anatomical details of the body. However, the anatomical details have not been well studied in *Macaca fuscata*. Arterial models could be one of the anatomical bases for the phylogenetic and functional differences among species, since the arterial supply could be associated with the muscular performance, especially locomotor behaviour. In this study, five thoracic limbs of *Macaca fuscata* adults were dissected to analyse the vessels. Patterns of arterial distribution in the thoracic limbs of *Macaca fuscata* were compared with those in other primates. The results indicated that the arterial distribution in the Japanese monkeys was more similar to those in *Macaca mulatta* and *Papio anubis*, which is consistent with phylogenetic similarities. However, compared with *Papio anubis* and other macaques, there were anatomical differences in several points, including (1) the origin of the common, anterior, posterior circumflex, and profunda brachii, and (2) the origins of the collateralis ulnaris artery. The comparative anatomy of the arteries in the forelimb of *Macaca fuscata*, along with the anatomical studies in other primates, indicated characteristic patterns of brachial artery division and the number of the palmar arches in primates, which is consistent with the phylogenetic division among New World primates, Old World primates, and apes.

## 1. Introduction

Japanese monkeys (*Macaca fuscata*) have been used as experimental animals in physiological studies and in many other studies on their ecology, zoology, and behaviour [1–4]. However, there are very few anatomical studies on *Macaca fuscata*. In general, *Macaca fuscata* display some behavioural characteristics compared with other primates of the genera *Macaca* because of their geographical isolation (i.e., they are strictly Japanese, they show different positional behaviour of free ranging, and in ecological aspects, they are more arboreal than other genera of macaques, specifically compared with the rhesus). Furthermore, they show other specific behaviours, such as heating their bodies in hot water spas in winter, fur colour [5], and anatomical differences in some arm muscles compared with the rhesus [6]. These characteristics could be explained by anatomical characteristics [3].

In addition to morphological similarities, biochemical and behavioural characteristics could help to identify taxonomic groups. However, more studies are required in primatology [7], especially studies on the basic anatomy of the group *Macaca*, in which previous studies focused mainly on *Macaca mulatta* in an ancient book [8], in some specific papers [9–17], or in comparative studies on vessels [18–20].

Some characteristics of *Sapajus* among primate species/genera could be explained by anatomical details [21–24]. *M. fuscata* displays characteristic behaviours such as stone handling [4], locomotor behaviour, gait position, and intermittent bipedalism, which could be explained by detailed anatomical studies. It is common that behavioural studies are carried out without anatomical bases. These studies sometimes, due to the absence of morphological bases, result in incorrect functional/behavioural interpretations [21, 23–25].

Scientific literature on the anatomy of *M. fuscata* anatomy is very limited [6]. On the other hand, comparative anatomical studies among primate species could improve phylogenetic and evolutionary knowledge [7], provide new data for new knowledge on the species, and, at least, support the proximity or reveal phylogenetic and taxonomic distance among taxa. As a whole, anatomical studies have focused mainly on muscles and bones for supporting phylogenetic and taxonomic data. Nevertheless, some recent investigations suggest the arterial supply as a physiological basis for muscle action, gait position, and tool use; so, putatively, arterial patterns could be used as a secondary analysis in comparative anatomy among primates as anatomical bases of such taxonomy, evolutionary comparison, and, in a specific and deep analyses, some behaviours [25–29].

Although the arteries present some variations in different individuals of the same species and laterality in the same area [30, 31], a tentative pattern could not be established. For instance, in the forelimb of primates, the absence or division of the distal part of the brachial artery into the radialis and ulnaris arteries is observed, which is dependent on primate species [26–28, 30, 32]. Apes have two palmar arches, which could be an exception in the *Gorilla* according to Sonntag [33], while the other primates have only one arch, which is the superficial one [28, 30, 32].

Indeed, these patterns are well-established in arterial anatomy. Thus, arterial models of arteries could be, at least as support for muscle and bone studies, one of the anatomical ways to characterize the differences among species, not only in phylogenetic but also in functional terms, since the arterial supply could be associated with muscular performance, especially in locomotor behaviours [25, 29].

Hypothetically, the anatomical data of the forelimb arteries in *M. fuscata* could be similar to those in the genera *Macaca* and *Papio* due to their phylogenetic proximity, i.e., subfamily Cercopithecinae [7].

Accordingly, the arterial anatomical model of *M. fuscata* should be examined, since as far as we know, the arterial model of the forelimb arteries of *M. fuscata* have not been reported previously.

Therefore, we examined the anatomy of the arteries in the forelimb of *M. fuscata*, described their distributions (origins and branches), and finally proposed a hypothetical theoretical explanation for an arterial model in *M. fuscata* to be compared with those in other primates, including New World primates (*Sapajus libidinosus* [26–28], *Saguinus leucopus* [34], *Callimico goeldii* [35]), *M. mulatta*, and *P. anubis* [18, 19, 30], all apes [18, 19, 30, 32], and modern humans [30, 32]. Finally, we discussed whether the arterial patterns in the forelimb might be used to distinguish primate groups, and whether their variations among the groups might be associated with physiological and behavioural characteristics.

## 2. Materials

### 2.1. Samples

Five thoracic limbs of *M. fuscata* adults were dissected at the Laboratory of System Emotional Science, Graduate School of Medicine, and Pharmaceutical Sciences, University of Toyama, Japan. Nine adult *S. libidinosus* specimens (three females and six males) were used to check other previous publications about these primates [21–23, 25–29], in a total of 18 limbs. Their weights were between 1 and 4 kg. No animal was killed for the purposes of this study; five of them suffered accidental deaths in their natural habitats and were deposited in the anatomical collection of the Museum of Morphology at the Federal University of Tocantins, Tocantins State, Brazil. The other four belonged to the Brazilian Institute of Environment and Renewable Natural Resources (IBAMA) archive and were donated for studies in the 1970s. Both forelimbs of all *S. libidinosus* previously dissected were analysed for the purpose of this work, which was approved by the Institutional Ethical Committee from the Federal University of Goiás, Goiás State, Brazil (CoEP-UFG 81/2008, authorization from the IBAMA number 15275).

### 2.2. Preparation of Animals for Dissection

The dead bodies/pieces were provided by the Primate Research Institute at Kyoto University, Kyoto, Japan. In a complete body, both forelimbs were dissected plus three more separated limbs, two right, and one left, totalizing 5 forelimbs, 2 right, and 3 left ones. These animals suffered a natural death in the Primate Research Institute at Kyoto University. One complete body and three forelimbs were kept frozen, and afterward, they were sent to Toyama University where they were placed in boxes and immersed in 10% formaldehyde, as for *S. libidinosus*.

### 2.3. Dissection and Documentation

The forelimbs of *M. fuscata* were dissected and *S. libidinosus* was studied, with an emphasis on arteries, and photographed with a digital camera (Canon SX610 HS). For the other primates, the data were obtained from literature mainly from Manners-Smith [18–20] for New World primates, *Papio* and *M. mulatta*; Swindler and Wood [30] for *Papio*, *Pan*, and modern humans; Gibbs [32] for all apes; and Standring [31] for modern humans. The arterial nomenclature was based on Nomina Anatomica Veterinaria (NAV) [36].

## 3. Results and Discussion

The arterial model for the five thoracic limbs of *M. fuscata* was quite similar, permitting a unique description of these animals. The few differences were commented on in the general discussion just for one separated limb, i.e., for 20% of the limbs. Remarkable differences were not observed in the right and left forelimbs of the same animal. The running and vascular irrigation of each specific artery was described in comparison with other primates.

### 3.1. Axillary Artery

In *M. fuscata*, the axillary artery is the continuation of the subclavian artery gives off the subscapularis, circumflexa scapulae, circumflexa humeri, and thoracodorsalis arteries in the arm and continues as the brachial artery (Table 1, Figure 1). The origin at the subclavian artery and continuation as the brachial artery is a common pattern in *C. goeldii*, *S. libidinosus*, *M. mulatta*, *P. anubis*, apes (*Pan troglodytes*, *Gorilla gorilla*, *Pongo pygmaeus*, and *Hylobates lar*), and modern humans [18, 26, 32, 35]. The emitted branches are similar to those in *S. libidinosus*, *P. troglodytes*, *G. gorilla*, *Pongo pygmaeus*, *H. lar*, and humans. However, in *M. mulatta*, the axillary artery was reported to emit branches including the circumflexa humeri, profunda brachii, collateralis radialis, and collateralis ulnaris [18], and in *P. Anubis*, the branches are collateralis media, profunda brachii, collateralis ulnaris, circumflexa humeri cranialis and caudalis, and brachialis [32] (Table 1, Figure 1). In *C. goeldii*, a short trunk was observed, which forms the thoracoacromialis and thoracic lateralis arteries [35].

The branches of the axillary artery, in four of the five limbs (80%) used in this study, displayed important differences from other primates. In *M. fuscata*, the subscapularis artery emerged from the axillary artery, and it did not emit the collateralis ulnaris and radialis arteries, as in *P. anubis* and *M. mulatta* (Table 1, Figure 1, Figure 2).

### 3.2. Brachialis Artery

The axillary artery gives off the brachial artery in *M. fuscata*, as well as in *C. goeldii*, *S. libidinosus*, *M. mulatta*, *P. anubis*, all apes, and modern humans [18, 26, 30, 32, 35]. An important point is that the brachialis can be short or absent in *S. libidinosus* (for more details, see [26]), which is similar to *C. goeldii* [35]. The emitted branches observed in *M. mulatta* from the brachialis artery are the profunda brachii, collateralis ulnaris, radialis, and ulnaris arteries. Except for *S. libidinosus*, the similar emitted rami from the brachial artery in other studied primates are the profunda brachii, radialis, and ulnaris arteries [18, 27, 32]. According to Manners-Smith [18–20], the brachialis superficialis is the name of radialis artery in the arm, which is the name used by Hill for *C. goeldii* [35].

In detail, the brachialis artery gives off, in *P. anubis* and *M. mulatta*, the profunda brachii, collateralis ulnaris, radialis, ulnaris, brachialis superficialis, and interossea communis arteries [18], and only in *P. anubis*, the other branches are the dorsalis ramus of recurrens ulnaris, cranialis and caudalis interossea, and antebrachialis superficialis (as a superficial part of the radial), giving off both recurrens ulnaris [19]. In apes, the emitted branches are the profunda brachii, nutricia humeri (specifically for *Gorilla*), collateralis ulnaris, radialis, ulnaris, recurrens ulnaris dorsalis, and palmaris rami (as a variant from a common trunk in 50% of *P. troglodytes* and Asian apes), interossea communis (*P. troglodytes*), interossea cranialis (for 33% of *P. troglodytes*), and interossea caudalis (*Pan paniscus*, *G. gorilla*, *Pongo pygmaeus*, and *H. lar*) [32].

In modern humans, the brachialis artery branches are the profunda brachii, nutricia humeri, collateralis ulnaris, radialis, ulnaris, recurrens ulnaris dorsalis (and palmaris rami (as a variant)), and interossea communis arteries [32] (Table 1, Figure 1, Figure 2).

Differently from other primates, the brachialis artery does not emit the interossea communis in *M. fuscata* observed in this work, but the ulnaris artery gives off the interossea communis (Table 1, Figure 3).

### 3.3. Subscapularis Artery

The subscapularis artery originates from the axillary artery together with the circumflex humeri caudalis and cranialis rami and thoracodorsalis arteries in *M. fuscata* (Table 1, Figure 1). This artery, which is absent in *S. libidinosus* [26], originates from the axillary artery in a common trunk with circumflexa scapulae in *P. anubis* [30], from the communis circumflexa in *P. troglodytes* and *Hylobates lar* [32] or from the axillary artery in a common trunk with the circumflexa scapulae and circumflexa humeri cranialis in *P. troglodytes* [30]. In modern humans, the subscapularis artery is the largest branch of the axillary artery and emits the circumflexa scapulae artery [37].

In *P. anubis* [30] and all apes [30, 32], the branches of the subscapularis artery have not been reported, because it originates in common with the circumflexa scapulae that is the final branch of the subscapularis artery in modern humans [37].

The subscapularis artery in *M. fuscata* displays a distribution similar to *P. anubis* (Table 1, Figure 3, Figure 2).

### 3.4. Circumflexa Humeri Cranialis and Caudalis and Related Arteries

The circumflexa humeri cranialis and caudalis arteries originate from the subscapularis artery. In one case, it emits the profunda brachii (Figure 1(b)) in the arm of *M. fuscata*. In general, these features of the circumflexa humeri cranialis and caudalis arteries are identical to other primates cited here [18, 27, 30, 32], except its origins in *S. libidinosus* [27] and *Pongo pygmaeus* [18] and emitted branches in African apes (*P. troglodytes* and *G. gorilla*) and *H. lar* [32] (Table 1, Figure 1, Figure 2). In *C. goeldii*, the axillary artery emits a large trunk that is the origin of the subscapularis and collateralis radialis arteries [35]. In *S. libidinosus*, the circumflexa communis artery can originate from the axillary, radialis, or from a big trunk in common with other arteries of the arm [27]. In *Pongo pygmaeus*, this artery also originates from a common trunk with the profunda brachii [18] and emits the profunda brachii in *P. troglodytes* and Asian apes (*Pan paniscus*, *Pongo pygmaeus*, and *H. lar*), the circumflexa scapulae in African apes (*P. troglodytes* and *G. gorilla*) and *H. lar*, and the subscapularis in *P. troglodytes* and *H. lar* [32].

Identically to *M. mulatta*, the circumflexa humeri emit only both circumflexa humeri cranialis and caudalis in *M. fuscata*, which is different from all apes where the profunda brachii could be a ramus from the trunk of the circumflexa humeri (Table 1, Figure 1). The circumflexa humeri cranialis artery is a final branch and originates from the axillary artery in *P. anubis* [18] and humans [32] and from the circumflexa humeri trunk in *M. fuscata*, *S. libidinosus* [27], all apes, and modern humans [32]. The circumflexa humeri caudalis artery is a final branch in *M. fuscata* and all other primates cited here, which is similar to the circumflexa humeri cranialis. It originates from the axillary artery in *P. anubis* [18] and modern humans [32] and from the trunk of the circumflexa humeri in *M. fuscata*, *S. libidinosus* [27], all apes, and modern humans, where the circumflexa humeri caudalis artery originates from the profunda brachii artery as a variant [32] (Table 1, Figure 1, Figure 2). The distribution of both the circumflexa humeri arteries in the humerus and their origin are similar for all primates, except for *P. anubis*, where they originate from the axillary artery (Table 1, Figure 1, Figure 2).

In *M. fuscata*, the profunda brachii artery originates from the brachialis artery (or from the trunk of the circumflex humeri arteries in one case (20%) and emits the collateralis radialis artery (Table 1, Figure 1, Figure 2), but the radialis proximalis was not found in the limbs of *M. fuscata* in this work. In *C. goeldii*, the profunda brachii originates from the brachial artery and through the supracondylar foramen [35]. In *S. libidinosus*, the profunda brachii originates from the ulnaris artery [27], from the axillary or brachial artery in *M. mulatta* or *P. anubis* [18], from the axillary or brachialis artery in 67% of *P. troglodytes* and sometimes in *H. lar*, from a common trunk with the axillary artery in *Pongo*, and from the brachialis artery in modern humans [32]. Hill cites the collateralis radialis artery with the same description of the profunda brachii for *C. goeldii* [35], which originated from the brachial artery; in *M. fuscata*, the collateralis radialis originates from brachialis artery as the most of primates studied (see below).

In other primates studied here, the profunda brachii gives off the collateralis radialis artery in *S. libidinosus* [27]; collateralis ulnaris, collateralis radialis, and collateralis media in *M. mulatta* and *P. anubis*; the collateralis radialis and collateralis media in all apes; and the collateralis radialis and collateralis media arteries, as separate branches in modern humans [30]. The branch from the profunda brachii commonly found in all the primates studied here is the collateralis radialis artery. However, the collateralis media artery was not found in *M. fuscata*, and an origin of the collateralis radialis at the circumflexa humeri trunk artery was found in one case (20%).

### 3.5. Collateralis Ulnaris and Radialis Arteries

The brachial artery gives off the collateralis radialis artery that is a final muscular branch in *M. fuscata* (Table 1, Figure 1(c)), except for 1 case (20%) (Figure 1(a)), it originates from profunda brachii artery. In *S. libidinosus*, the collateralis radialis originates from the radialis directly, from a common trunk with the caudal part of the collateralis radialis artery, from the ulnaris artery infrequently, and from the rete articulare cubiti [27]. In *P. anubis*, it originates from the axillary artery [18]; in African apes, the collateralis radialis originates from the brachial artery; in Asian apes, it originates from the profunda brachii [32]; and in modern humans, it originates from the brachial artery or from the profunda brachii as a variant [32]. The collateralis radialis artery is a final branch in *P. anubis*, all apes, and modern humans [18, 30, 32]. The origin of the collateralis radialis artery is identical for all primates, except *P. anubis*, where the origin is the axillary artery (Table 1, Figure 1, Figure 2).

The collateralis ulnaris artery is a final branch and originates from the brachialis artery in *M. fuscata*. It is a final branch in *M. mulatta*, *P. anubis*, all apes, and modern humans [18, 27, 32], and it originates from the brachial artery in all apes and modern humans [32] and from the brachialis or brachialis superficial (this name was used by Manners-Smith [18] and Hill [35] and corresponds to the radialis artery) in *M. mulatta* and *P. anubis* [18]. In *S. libidinosus*, the cranialis part of the collateralis ulnaris artery originates from the radialis directly or in a common trunk with the collateralis ulnaris artery, from the ulnaris artery infrequently, and from the rete articulare cubiti [27]. The origin of the caudalis part of the collateralis ulnaris artery is identical in all the primates studied here, but in *P. anubis* and *M. mulatta*, the radialis artery could emit it (Table 1, Figure 2).

### 3.6. Radialis and Ulnaris Arteries

The radialis artery originates from the brachialis artery and emits the recurrens radialis, ramus carpeus dorsalis, ramus dorsalis for the pollicis (princeps pollicis), digitales for second digiti (index artery), arcus palmaris superficialis, and interossea communis together with the ulnaris in *M. fuscata* (Table 1; Figures 2, 3, 4, 5 and 6). In *S. libidinosus*, the radialis artery originates from the axillary artery (or infrequently from the brachialis artery) and gives off the collateralis ulnaris, recurrens radialis [27], and ramus carpeus dorsalis [38]. The radialis artery originates from the brachialis artery in *P. anubis*, *M. mulatta* [18], apes (*Pan paniscus*, *G. gorilla*, *Pongo pygmaeus*, and *H. lar*), and modern humans [32], and in *C. goeldii*, it is called the superficialis brachialis [35]. It gives off the recurrens radialis, ramus carpeus dorsalis, metacarpae dorsalis, perforans branches and digitalis, and ramus carpeus palmaris, which emits the ramus superficialis palmaris to the arcus palmaris superficialis in *M. mulatta* and *P. anubis* [19].

The radialis artery emits the ramus dorsalis for the pollicis in *Pan paniscus*, *G. gorilla*, *Pongo pygmaeus*, and *H. lar* and emits the recurrens radialis in 33% of *P. troglodytes*. It emits the recurrens palmaris and ramus palmaris superficialis in all apes, except for G. *gorilla.* However, the radialis artery may be absent in *H. lar*.

The radialis artery emits the carpeus dorsalis, ramus dorsalis for the pollicis, ramus digitalis, arcus palmaris profundus, rete carpi dorsale, a branch for arcus palmaris superficialis, and ramus carpeus palmaris arteries in *P. troglodytes* [32].

In modern humans, the radialis artery emits the recurrens radialis, recurrens ulnaris, arcus palmaris superficialis, ramus carpeus dorsalis, ramus dorsalis for the pollicis, and digitales for second digiti (index artery) [32].

The origin of the radialis artery is identical in all the primates studied here, except for some cases of *S. libidinosus* [28]. However, the differences are found in terms of its contribution to formation of the arcus palmaris. In *Pan paniscus*, *G. gorilla*, *Pongo pygmaeus*, and *H. lar*, the radialis artery emits branches for the arcus palmaris superficialis [32], while it emits only a branch for the arcus palmaris superficialis in *P. anubis*, *M. mulatta*, and *M. fuscata*.

The ulnaris artery in *M. fuscata* originates from the brachialis artery and emits the recurrens ulnaris, the interossea communis together with the radialis, arcus palmaris superficialis, and ramus carpeus palmaris (Table 1, Figure 3, Figure 4, Figure 2). According to Hill [35], the ulnaris artery is a continuation of the profunda brachii artery for *C. goeldii*. In *S. libidinosus*, the ulnaris artery originates from the axillary or infrequently from the brachialis artery and gives off the collateralis ulnaris (occasionally), collateralis media, collateralis radialis [27], interossea communis, recurrens ulnaris, arcus palmaris superficialis, and ramus dorsalis for the pollicis (princeps pollicis) [38]. It goes through the supracondylar foramen in *S. libidinosus* [27] and *S. leucopus* [7, 34], and it similarly occurs in cats [34, 39]. The ulnaris artery originates from the brachialis artery in *P. anubis*, *M. mulatta* [18], *Pan paniscus*, *G. gorilla*, *Pongo pygmaeus*, *H. lar*, and modern humans [32], while it gives off the arcus palmaris superficialis a fine ramus carpeus dorsalis in *P. anubis* [19].

The ulnaris artery emits the ramus dorsalis for the pollicis (princeps pollicis) in *G. gorilla* and Asian apes; digitales for second digiti (index artery) and ramus carpeus dorsalis in *G. gorilla* and *Pongo pygmaeus*; contributes to the arcus palmaris superficialis and profundus, interossea communi in *P. troglodytes*; and the interossea cranialis, ramus carpeus dorsalis, ramus carpeus palmaris, arcus palmaris superficialis, and profundus in all apes and modern humans [32].

In modern humans, the ulnaris artery emits the recurrens ulnaris, interossea communis, ramus carpeus dorsalis, ramus carpeus palmaris, and arcus palmaris profundus [32].

Except for most *S. libidinosus*, the ulnaris artery originates from the brachialis artery in all primates studied here [28, 30–32], and it is the main source of the arcus palmaris superficialis and profundus for most of the primates in this work, except *P. anubis* [30], *M. mulatta*, and *M. fuscata*, where the radialis artery has a more important or identical role in the superficial palmar arch. Interestingly, the interossea communis originates from an anastomosis of both ulnaris and radialis arteries, as a case not cited for the other primates studied here (Table 1, Figure 3, Figure 4, Figure 2).

### 3.7. Arcus Palmaris

The arcus palmaris profundus is absent in *M. fuscata*, *C. goeldii* [35], *S. libidinosus* [38], *M. mulatta*, and *P. anubis* [19] and is very fine in *Pongo pygmaeus* [32] (Figure 7, Figure 8). In all apes, the arcus palmaris profundus is formed by the ramus palmaris profundus of the ulnaris artery and completed by the radialis or by the ramus dorsalis for the pollicis (princeps pollicis) in African apes or by the digitales for second digiti (index artery) in 50% of *Pongo pygmaeus* [32]. In modern humans, it is formed by the arcus palmaris profundus of the ulnaris artery and completed by the radialis [32]. In *G. gorilla*, *H. lar*, and modern humans, the arcus palmaris profundus gives off the metacarpae palmaris rami [32].

In *M. fuscata*, the arcus palmaris superficialis originates in part from the ulnaris and in part from the radialis arteries and emits the digitalis palmaris communis rami (Table 1, Figure 7, Figure 2). The radialis artery is the principal component of this arch, which is similar to *M. mulatta* and *P. anubis* [19].

The ulnaris artery gives off the arcus palmaris superficialis, which is completed by the radialis in *S. libidinosus*, and emits the digitalis palmaris communis rami in *S. libidinosus* [38]. A unique palmar arch originating from the ulnaris artery is cited for *C. goeldii* [35]. In *M. mulatta* and *P. anubis*, it is formed by a small branch of the ulnaris and radialis arteries and emits the digitalis palmaris communis rami and princeps pollicis [19]. In all apes, the arcus palmaris superficialis originates from the ulnaris artery, ramus palmaris superficialis of the radialis, is completed by the radialis artery or princeps pollicis in 50% of *H. lar*, and emits the digitalis palmaris propriae arteries in modern humans [32]. In modern humans, the arcus palmaris superficialis is formed by the ulnaris and is completed by the superficial ramus palmaris superficialis of the radialis and rarely by the princeps pollicis [32].

## 4. General Discussion

### 4.1. Structure of the Brachialis Artery in Primates

The brachialis artery has a remarkable difference, specifically its size, in the forelimb arteries among primates, additionally, the axillary artery in *P. paniscus* present very different organization in relation to modern humans [40]. The radialis and ulnaris arteries originate directly from the axillary artery in *S. libidinosus* because of the absence or presence of a small brachialis [18, 26], as also occurs with *C. goeldii* [35] and *Galago senegalensis* [41], and from the brachialis approximately in the distal two-thirds of the humerus in other New World primates studied by Manners-Smith [18, 19] (e.g., the genera *Lagothrix* and *Saimiri* that receive the identical description and designation of arteries of the arm given for Cebidae [19, 42]). Except for *Lagothrix* [7, 19, 42], the ulnaris artery, or the brachialis profunda (as it is called by Manners-Smith), runs in parallel together with the medianus nerve across the supracondylar foramen [19, 42].

The presence of the supracondylar foramen with the medianus nerve and ulnaris artery coursing through it was cited for *Saimiri* [7, 19], *Sapajus* [7, 19, 27], *S. leucopus* [7, 34], and *C. goeldii* [35] in the New World primates and in the *Nycticebus* [19] and most of the living prosimians [7]. Usually this foramen is not found in *Cebuella*, *Callitrix*, *Ateles*, *Allouata*, and *Callicebus* [7]. Interestingly, for other domestic mammals, the supracondylar foramen, where the medianus nerve and brachialis artery pass through it, is cited only for cats [39].

Despite Ankel-Simons [7] citing that the supracondylar foramen (called the entepicondylar foramen by this author) is derived from archaic mammals, no explanation for the phylogenetic correspondence seems to exist among New World primates and prosimians [43] with the genus *Felis* in relation to the existence of this feature and the reason for derivative primates (i.e., Old World primates and apes) do not present with this characteristic.

If the supracondylar foramen could generate bone protection for a medianus nerve and ulnaris/brachialis artery in a fragile position (e.g., where they are more superficial), maybe because the modifications of the curvature of the forelimbs bones in the evolution [44], however, the absence of this foramen seems more dubious in continuation of evolution. A detailed evolutionary study could be performed in this sense.

In *P. anubis* [30] and *M. mulatta* [19], the brachialis artery divides into the radialis and ulnaris arteries at a point on the humerus one-third proximal from the elbow joint, which is identical to the pattern in *M. fuscata*. In *P. troglodytes*, the brachialis divides more distally than in *P. anubis* [30] and *M. mulatta*. In all apes, the brachialis divides at the level of the elbow joint [30], and in modern humans, it divides below the elbow joint [37]. Thus, the more recent the evolutionary group is, the longer the brachialis.

The anatomy of the brachial division seems to coincide with primate evolution, since primate evolution is associated with the descent from the trees [45] and also coincides with the presence/absence of the structure of the arcus palmaris.

Indeed, the morphological structure of the arcus palmaris and size of brachial artery size should be taken into consideration for a more detailed analysis of the vascularization of the forelimb in primates, since the size of the brachialis artery is associated with the structure of the arcus palmaris. New World and Old-World primates display proximal division from the brachial artery and have the presence of one palmar arch, while apes and modern humans display division of the brachial artery around the elbow fossa and have two palmar arches. For example, it is possible that larger blood pressure drops in the branches (radialis and ulnaris arteries) would permit only one palmar arch in New World primates. Further, detailed simulation of blood flow will be required based on the actual sizes of the brachialis, radialis, and ulnaris arteries, as well as palmar arches. Indeed, the fact of the crown hominoids possibly to abduct the arm above the shoulder indicates a need for more accurate biophysical studies about the blood flux in the vessels of the primates [46].

### 4.2. Forelimb Arterial Pattern in Primates

The vessels displayed a very unsteady arrangement across individuals and different antimeres in the same individual, which is more often observed in veins [30]. This is probably one of the reasons why few studies have investigated vessels in relation to evolution. Comparative primate studies on the hindlimb vessels were performed in relation to bipedalism and bipedal gait and reported different arterial patterns among primates for the pelvis and hindlimbs of *Sapajus* [23, 25].

An interesting case of different distribution cited here occurs in Lorisiformes, that is the existence of a vascular bundles of the main artery generating 50 small ones.

Here, we present three different models of arteries in the upper limbs of primates with regard to the height of the brachial division which may be associated with locomotor behaviour and taxonomy.

The first model presents an absent or short brachial artery with one palmar arch, which is observed in monkeys with arboreal locomotion (Figure 8, left panel), such as New World primates [18–20, 27] and Lorisiformes [43], not shown here. In the second model, the brachialis divides at a point on the humerus approximately one-third proximal from the elbow joint, where only one palmar arch is observed. Old World primates with arboreal locomotion are general examples of this second model (Figure 8, middle panel). The description of forelimb arteries with this pattern has been reported in *M. mulatta* [19] and, now, for *M. fuscata* in this work. The third model refers to apes and modern humans with more terrestrial locomotion that display more distal division of the brachialis artery and the existence of two palmar arches in the arcus palmaris (Figure 8, right panel), except for *Pongo pygmaeus*.

Hypothetical inference of the relationships between the morphological differences in arterial models and primate evolution is noted above. These models might provide anatomical support for taxonomy division into New World primates, Old World primates, apes, and modern humans with evolutionary and behavioural studies.

An interesting study could be performed using the hominoids, despite the difficulties of interpretation due to the shortage of complete bodies.

Additionally, a possible problem with tentative of the solution here was about the ancient nomenclature of the forelimb arteries, the authors of the early 20^th^ century [18–20, 35, 41, 42], starting by Manners-Smith [18–20], gave name for arteries according to the region of the forelimb, i.e., they avoided gave the name ulnaris and radialis in the arm. In this way, the hodiern names as ulnar artery was called profunda brachii; the radialis called superficialis brachialis artery and hodiern name of profunda brachii was called radialis collateralis artery. However, as the descriptions are identical, then we follow the nomenclature of modern authors [30, 32] and of the NAV [36] (Table 2).

## 5. Conclusions

Comparative studies provide important data with evolutionary, behavioural, phylogenetic, and taxonomic ramifications [7, 47] and should be performed constantly to promote such interdisciplinary studies. However, anatomical studies on primates are scarce, specifically those on arteries. The available information on the anatomy of primate vessels is restricted to the work of Manners-Smith [18, 19] and Bang [42], an old study on the anatomy of apes performed as a thesis [32], a few books, and sparse papers.

The present study indicated that the overall arterial distribution in *M. fuscata* was similar to *M. mulatta* and *P. anubis*. However, some differences were observed, including (1) the origin of the common, cranial, caudal circumflexa, and profunda brachii and (2) origins of the collateralis ulnaris arteries in *M. fuscata* were different from those in *P. anubis* and other macaques.

Second, the comparative anatomy of the arteries in the forelimb of *M. fuscata* proposed the three arterial patterns in the forelimb in terms of length of the brachial artery and number of palmar arches in the arcus palmaris. These data led to a taxonomy confirmation of the differences of classification of the groups of New World primates, Old World primates, and apes.

## Figures and Tables

**Figure 1:** Medial view of the shoulder and proximal part of the arm in Macaca fuscata. (a) Common pattern found in M. fuscata. (b) A variation of the distribution of the proximal arteries in the arm. The main difference is the origin of the profunda brachii from the brachial in (a) and from the common circumflexa humeri artery in (b). (c) A variation of the collateralis radialis artery; originates from the profunda brachii artery in (a) and from the brachialis artery in (c). (1) Axillary artery; (2) Circumflexa humeri communis, subscapularis, circumflexa scapulae, and thoracodorsalis; (3) Common trunk for the subscapularis, circumflexa scapulae, and thoracodorsalis; (4) Circumflexa humeri communis; (5) Thoracodorsalis; (6) Circumflexa scapulae; (7) Subscapularis; (8) Circumflexa humeri cranialis; (9) Profunda brachii; (10) Brachialis; (11) Collateralis ulnaris; (12) Collateralis radialis, white arrow indicates the same artery of 12, but with normal origin from the brachialis artery, ^∗^ muscular branch. The head black arrow indicates the circumflexa humeri caudalis. Name of muscles: (I) Coracobrachialis, (II) Biceps brachii caput brevis, (III) Triceps brachii caput mediale, (IV) Teres major, (V) Tendon of latissimus dorsi, (VI) Subscapularis.

**Figure 2:** Schema of the common arterial pattern in the thoracic limb of Macaca fuscata. (1) Axillary artery; (2) Subscapularis artery and its branches: interossea communis, subscapularis, circumflexa scapulae, and thoracodorsalis; (3) Common trunk for subscapularis, circumflexa scapulae, and thoracodorsalis; (4) Common circumflexa humeri; (5) Thoracodorsalis; (6) Circumflexa scapulae; (7) Subscapularis continuation; (8) Circumflexa humeri cranialis; (9) Profunda brachii; (10) Brachialis; (11) Collateralis ulnaris; (13) Radialis; (14) Ulnaris; (15) Recurrens ulnaris; (16) Recurrens radialis; (17) Interossea communis; (25) Arcus palmaris superficialis; (26) Princeps pollicis; (∆) Digitales communis arteries; (27) Collateralis ulnaris; (28) Interossea cranialis; (29) Interossea caudalis. An arrow indicates the circumflexa humeri caudalis.

**Figure 3:** Medial view of the right elbow in Macaca fuscata. (13) Radialis artery, (14) Ulnaris artery, (15) Recurrens ulnaris, (16) Recurrens radialis, (17) Interossea communis, (17a) contribution from radialis artery, (17b) contribution from ulnaris artery. Muscles: (I) Tendon of brachialis, (II) Biceps brachii, (III) Triceps brachii caput mediale, (VII) Flexor carpi ulnaris, (VIII) Brachioradialis, (ø) median nerve.

**Figure 4:** Caudal view of the distal forearm in Macaca fuscata, right forelimb. (18) Superficial branch of the radialis artery, (19) Deep branch of the radialis artery, (20) Ulnaris artery profundus ramus, (21) Superficial branch of the ulnaris artery. Muscles: (IX) Brachioradialis, (X) Tendon of palmaris longus. (XI) Flexor carpi ulnaris tendo, (XII) Flexor digitorum superficialis, (XIII) Flexor carpi ulnaris tendon.

**Figure 5:** Medial view of the carpus in Macaca fuscata. (22) Ramus carpeus dorsalis of the radialis artery, (*α*) Metacarpae dorsalis branches. Muscles: (XIII) Interossei (digitis II), (XIV) Extensor digiti I.

**Figure 6:** Dorsal view of the metacarpal region in Macaca fuscata. (22) Ramus carpeus dorsalis of the radialis artery, (23) Arcus metacarpae arch for radialis artery, (24) Arcus metacarpae from ulnaris artery, (*α*) Metacarpae dorsalis branches. Muscles: (XV) Extensor carpi radialis brevis, (XVI) Extensor digitorum communis tendon.

**Figure 7:** Palmar of the left hand of Macaca fuscata. (18) Ulnaris artery, (21) Radialis artery superficial ramus, (25) Arcus palmaris superficialis, (26) Princeps pollicis artery, (∆) Digitales communis arteries, (†) Communicating branches. Muscles: (ß) Interossei, (XVI) Abductor digiti I.

**Figure 8:** Schema of the arterial pattern in the right thoracic limbs in terms of division of the brachial artery and the number of the palmar arches.

**Table 1:** Comparative anatomy of the forelimb arteries of Japanese monkeys (this work), including *S. libidinosus* (New World primate), other *Macaca*, *P. anubis*, apes, and *Homo*. The previous studies were cited by the initials of the first authors with the species names. O: originates from; E: emits. References: MS1: Manners-Smith, 1910a; MS2: Manners-Smith, 1910b; SW: Swindler and Wood, 1973; G: Gibbs, 1999; AV1: Aversi-Ferreira et al., 2007a; AV2: Aversi-Ferreira et al., 2007b; AV3: Aversi-Ferreira, 2009.

Arteries/groups	*M. fuscata*		New World primate (*S. libidinosus*) (AV1, AV2, AV3)		*M. mulatta* and *P. anubis* (MS1, MS2)		All apes (G)		*Homo* (G)	
	O	E	O	E	O	E	O	E	O	E
Axillary (branches in the arm)	Subclavia	Common trunk for subscapularis, circumflexa humeri cranialis and caudalis, circumflexa scapulae, thoracodorsalis, brachial	Subclavia (AV1)	Radialis, ulnaris, circumflexa humeri cranialis and caudalis, brachialis (AV2)	Subclavia (MS1)	Profunda brachii, collateralis ulnaris, circumflexa humeri cranialis and caudalis, brachialis (*Papio*); circumflexa humeri cranialis and caudalis, profunda brachii, collateralis radialis, collateralis ulnaris cranialis part, (*Macaca*) (MS1)	Subclavia	Circumflexa humeri cranialis and caudalis, brachialis	Subclavia	Circumflexa humeri cranialis and caudalis, brachialis
Brachialis	Axillary	Profunda brachii, collateralis ulnaris, collateralis ulnaris caudalis part, radialis, ulnaris	Axillary or absent (AV2)	When present is a small branch and emits just radialis and ulnaris (AV2)	Axillary (MS1)	Profunda brachii, collateralis ulnaris, collateralis ulnaris caudalis part, radialis, ulnaris, brachialis superficialis, interossea communis (MS1), recurrens ulnaris dorsalis, cranialis and caudalis interossea, antebrachii superficialis (in *P. anubis* and one species of *Macaca*, in general, it is a superficial part of the radialis), gives off both recurrens ulnaris (*P. anubis*) (MS2)	Axillary	Profunda brachii, nutricia humeri (*Gorilla*), collateralis ulnaris, collateralis ulnaris caudalis part, radialis, ulnaris, cranialis and dorsalis ulnaris recurrens (as a variant, from a common trunk ½ *P. troglodytes* and Asian apes), interossea comumnis us (*P. troglodytes*), interossea cranialis us (1/3 *P. troglodytes*), interossea caudalis us (*Gorilla* and Asian apes)	Axillary	Profunda brachii, nutricia humeri, collateralis ulnaris, collateralis ulnaris caudalis part, radialis, ulnaris, cranialis and caudalis ulnaris recurrens (as a variant), interossea communis
Subscapularis	Axillary from a common trunk that generates other common trunk for circumflexa scapulae, thoracodorsalis and subscapularis	Cranialis and caudalis circumflex humeris, thoracodorsalis	Absent (AV1)		Axillary in a common trunk with circumflexa scapulae in *P. anubis* (SW)		Cranialis and caudalis circumflex humeris, in *P. troglodytes* and *Hylobates lar* (G). Axillary in a common trunk with circumflexa scapulae and circumflexa humeri cranialis in *P. troglodytes* (SW)		Axillary (Gray, 1918)	Circumflexa scapulae (Gray, 1918)
Circumflexa humeri cranialis and caudalis	Common trunk with other trunk for circumflexa scapulae, thoracodorsalis and subscapularis	Cranialis and caudalis circumflexa humeri	Axillary, radialis, in common with other arteries from a bigger trunk (AV2)	Cranialis and caudalis circumflexa humeri (AV2)	Axillary (*Macaca*) (MS1)	Cranialis and caudalis circumflexa humeri (*M. mulatta*) (MS1)	Axillary, a common trunk with the profunda brachii (*Pongo*) (MS1)	Cranialis and caudalis circumflexa humeri, profunda brachii (*P. troglodytes* and Asian apes), circumflexa scapulae (African apes and *H. lar*), subscapularis (*P. troglodytes* and *H. lar*)	Axillary	Cranialis and caudalis circumflexa humeri
Profunda brachii	Brachialis, circumflexa humeris (for one case)	Collateralis radialis	Ulnaris (AV2)	Collateralis radialis (AV2)	Axillary or brachialis (MS1)	Collateralis ulnaris, collateralis radialis, collateralis media (MS1)	Axillary, brachialis (2/3 *P. troglodytes*, sometimes in *H. lar*). Common trunk with axillary (*Pongo*) (MS1)	Collateralis radialis, collateralis media (MS1)	Brachialis	Collateralis radialis (MS1)
Collateralis ulnaris	Brachialis		Radialis directly or in a common trunk with collateralis ulnaris caudalis part, ulnaris (less frequently) (AV2)	Rete articulare cubit (AV2)	Axillary (*P. anubis*) (MS1)		Brachialis (African apes), profunda brachii (Asian apes)		Brachialis, profunda brachii (as variant)	
Caudalis part of the collateralis ulnaris	Brachialis		Radialis directly or in a common trunk with collateralis ulnaris, ulnaris (less frequently) (AV2)	Rete articulare cubit (AV2)	Brachialis or radialis (brachialis superficial) (MS1)		Brachialis		Brachialis	
Radialis	Brachialis	Recurrens radialis, interossea communis together with ulnaris, carpeus dorsalis, princeps pollicis, radialis index, arcus palmaris superficialis	Axillary, brachialis (less frequently) (AV2)	Collateralis ulnaris, recurrens radialis (AV2), carpeus dorsalis, (AV3)	Brachialis (MS1)	Recurrens radialis, ramus dorsalis (emits carpeus dorsalis and metacarpae dorsalis and perforans branches, index and ramus palmaris (emits the ramus palmaris superficialis to the arcus palmaris superficialis) (MS2)	Brachial	Dorsalis pollicis (*Gorilla* and Asian apes), recurrens radialis (1/3 *P. troglodytes*), recurrens palmaris, palmaris superficialis (except *Gorilla*, it may be absent in *H. lar*), carpeus dorsalis, princeps pollicis, index, arcus palmaris profundus (*P. troglodytes*), a branch for arcus palmaris profundus, carpeus palmaris (*P. troglodytes*), a branch for arcus palmaris superficialis	Brachial	Recurrens radialis, recurrens palmaris, palmaris superficialis, carpeus dorsalis, princeps pollicis,
Ulnaris	Brachial	Recurrens ulnaris, interossea communis interossea together radialis, arcus palmaris superficialis, ramus carpeus palmaris	Axillary, brachial (less frequently) (AV2)	Collateralis ulnaris (occasionally), collateralis media, collateralis radialis (AV2), interossea communis, recorrens ulnaris, arcus palmaris superficialis, princeps pollicis (AV3)	Brachialis (MS1)	Arcus palmaris superficialis, fine ramus carpeus palmaris, carpeus dorsalis (*P. anubis*) (MS2)	Brachialis	Dorsalis for the pollicis (*Gorilla* and Asian apes), (*Gorilla* and *Pongo*), metacarpae dorsalis (*Gorilla* and *Pongo*), contribute to superficialis and profundus palmaris arcus, interossea communis (*P. troglodytes*), interossea cranialis, carpeus dorsalis, carpeus palmaris, arcus palmaris profundus, arcus palmaris superficialis	Brachialis	Interossea communis, carpeus dorsalis, ramus carpeus palmaris, profundus and superficialis arcus palmaris
Arcus palmaris profundus	Absent	Absent	Absent [AV3]		Absent (MS2)		Very fine in *Pongo*, ramus palmaris profundus of the ulnaris, completed by the radialis, princeps pollicis (African apes), (1/2 *Pongo*)	Metacarpae palmaris (*Gorilla*, *H. lar*)	Arcus palmaris profundus of the ulnaris, completed by the radialis	Metacarpae palmaris
Arcus palmaris superficialis	Part from ulnaris and part from radialis	Metacarpae palmaris	Ulnaris (AV3)	Digitalis palmaris communis (AV3)	Ulnaris (smaller branch) and radialis (MS2)	Metacarpae palmaris, digitalis palmaris communis, princeps pollicis (MS2)	Ulnaris, ramus palmaris superficialis of the radialis, princeps pollicis (1/2 *H. lar*)	Digitalis palmaris communis	Ulnaris, completed by the palmaris superficialis ramus of the radialis, princeps pollicis (rare variation)	Digitalis palmaris communis

**Table 2:** Differences among the ancient and modern nomenclature for some arteries of the Primates' arm.

Primates	Nomenclature	
*C. goeldi* [35] *Galago senegalensis* [41] *Saimiri* [18–20] Cebidae (*Cebus/Sapajus)* [18–20] *L. lagothricha* [18–20, 42] *Papio anubis* [18–20] *Macaca mulatta* [18–20]	Former	Modern [30, 32, 36]
	Brachialis superficial	Radialis
	Collateralis Radialis	Profunda Brachii
	Profunda Brachii	Ulnaris

## Data Availability

All data are available upon request to the corresponding author (TAA-F).
